The article "Relationship between Circle of Willis Variations and Cerebral or Cervical Arteries Stenosis Investigated by Computer Tomography Angiography and Multitask Convolutional Neural Network" was published in 2021. Journal: J Healthc Eng.

# Relationship between Circle of Willis Variations and Cerebral or Cervical Arteries Stenosis Investigated by Computer Tomography Angiography and Multitask Convolutional Neural Network

**DOI:** 10.1155/2021/6024352

**Published:** 2021-10-31

**Authors:** Jin Hou, Ming Yong Gao, Ai Zhen Pan, Qiu Dian Wang, Bin Liu, Ya Bin Jin, Jia Bin Lu, Qing Yuan He, Xiao Dong Zhang, Wei Wang

**Affiliations:** ^1^Department of Radiology, The 2nd Affiliated Hospital of Guangzhou Medical University, Guangzhou 510260, China; ^2^Department of Radiology, Research Institute for Translation Medicine on Molecular Function and Artificial Intelligence Imaging, The First People's Hospital of Foshan, Foshan 528000, China; ^3^Center for Human Anatomy, School of Biomedical Sciences, University of Edinburgh, Edinburgh EH8 9XD, UK; ^4^Department of Interventional Medicine, The 2nd Hospital of Shandong University, Jinan 250033, China; ^5^Clinical Research Institute, The First People's Hospital of Foshan, Foshan 528000, China; ^6^Institute of Biomedical Engineering, Peking University Shenzhen Graduate School, Shenzhen 518055, China; ^7^Shenzhen Institutes of Advanced Technology, Chinese Academy of Sciences, Shenzhen 518055, China

## Abstract

Circle of Willis (CoW) is the most critical collateral pathway that supports the redistribution of blood supply in the brain. The variation of CoW is closely correlated with cerebral hemodynamic and cerebral vessel-related diseases. But what is responsible for CoW variation remains unclear. Moreover, the visual evaluation for CoW variation is highly time-consuming. In the present study, based on the computer tomography angiography (CTA) dataset from 255 patients, the correlation between the CoW variations with age, gender, and cerebral or cervical artery stenosis was investigated. A multitask convolutional neural network (CNN) was used to segment cerebral arteries automatically. The results showed the prevalence of variation of the anterior communicating artery (Aco) was higher in the normal senior group than in the normal young group and in females than in males. The changes in the prevalence of variations of individual segments were not demonstrated in the population with stenosis of the afferent and efferent arteries, so the critical factors for variation are related to genetic or physiological factors rather than pathological lesions. Using the multitask CNN model, complete cerebral and cervical arteries could be segmented and reconstructed in 120 seconds, and an average Dice coefficient of 78.2% was achieved. The segmentation accuracy for precommunicating part of anterior cerebral artery and posterior cerebral artery, the posterior communicating arteries, and Aco in CoW was 100%, 99.2%, 94%, and 69%, respectively. Artificial intelligence (AI) can be considered as an adjunct tool for detecting the CoW, particularly related to reducing workload and improving the accuracy of the visual evaluation. The study will serve as a basis for the following research to determine an individual's risk of stroke with the aid of AI.

The article "Relationship between Circle of Willis Variations and Cerebral or Cervical Arteries Stenosis Investigated by Computer Tomography Angiography and Multitask Convolutional Neural Network" was published in 2021. Journal: J Healthc Eng.

## 1. Introduction

Circle of Willis (CoW) is the most important collateral pathway to allow blood communication between the contralateral cerebral hemisphere and carotid-basilar artery, depending on the integrity of the anterior and posterior parts of the CoW. However, there are more than 20 types of variations in the CoW found commonly across populations. What is responsible for CoW variation remains unclear. Still, some researchers have demonstrated the relationships with cerebral and cervical diseases, such as cerebral ischemic stroke, aneurism, and white matter lesions [1–4]. Dissection was the initial avenue for CoW research, though now advanced mini- and noninvasive imaging techniques are used, including computer tomography angiography (CTA), magnetic resonance angiography (MRA), digital subtraction angiography (DSA), and transcranial Doppler ultrasonic. These techniques allow for in vivo observations of the CoW, enabling CoW research in both larger and more specific populations. MRA is a popular technique for being noninvasive and does not utilize iodine or ionizing radiation exposure. Still, MRA tends to overestimate the variation and stenosis, which is attributable to slow or turbulent flow in the stenosis lumen or thin segment [5]. CTA is a faster, more accurate examination than MRA, primarily since it can provide detailed information regarding the configuration of the CoW and the extracranial and intracranial arteries with one-stop scanning. In the study, using CTA data, the correlation between the variation in the CoW and factors, such as age, gender, and the stenosis of afferent or efferent arteries, were evaluated. At the same time, it was noted that visual evaluation for CoW variation would be highly time-consuming, likely taking more than 1 hour to delineate a complete cerebral and cervical artery, which is not impractical in clinical application. In recent years, computer-aided diagnosis has drawn much attention with the development of computer technologies, such as big data [6, 7] and deep learning [8]. It brings excellent progress in disease classification [9], anomaly detection [10, 11], and medical image segmentation [12, 13]. Automatic segmentation of cerebral vessels is required to perform automatic analysis of CoW variation. However, it is still challenging to segment cerebral arteries automatically due to the inhomogeneous intensity, complex topological shapes, vessel abnormality, and other complex features [14, 15]. Conventional methods segment vessels are based on low-level features with low accuracy and efficiency [16]. Here, we proposed a multitask CNN-based-cerebral artery segmentation method and validated its performance in our clinical datasets. The study will serve as a basis for the following research to determine an individual's risk of stroke with the aid of artificial intelligence (AI).

The article "Relationship between Circle of Willis Variations and Cerebral or Cervical Arteries Stenosis Investigated by Computer Tomography Angiography and Multitask Convolutional Neural Network" was published in 2021. Journal: J Healthc Eng.

## 2. Materials and Methods

### 2.1. Subjects

The study was approved by our institutional review board, and written informed consent was waived by the IRB due to the retrospective nature of the study. Between 2009 and 2019, the data from 15000 patients were retrospectively investigated, and CTA of cerebral or cervical arteries were analyzed by two independent radiologists. Some data were excluded if patients had encephalorrhagia, aneurysms, malignant tumors, and other diseases involving the arteries in the neck or the quality of images was not enough to analyze. Patients were selected and divided into six groups according to the age and the severity of cerebral or cervical artery stenosis: the young normal group (Yn), aged 21–35 years without stenosis of an artery; the senior normal group (Sn), aged 55–76 years without stenosis of an artery; the mild-moderate stenosis in afferent arteries group (AMs), with mild or moderate stenosis of the common carotid artery (CCA), internal carotid artery (ICA), or basilar artery (BA) but without simultaneous severe stenosis of bilateral vertebral artery (VA); the severe stenosis in afferent arteries group (ASs), with severe stenosis of the CCA, ICA, BA, or both VA; the severe stenosis of efferent arteries group (ESs), with severe stenosis of postcommunicating parts of an anterior cerebral artery, middle cerebral artery, or posterior cerebral artery (pACA, pMCA, or pPCA); and the control group of efferent arteries (Ec), with normal postcommunicating parts and normal or middle stenosis of afferent arteries.

### 2.2. CT and CT Angiography

Using the scanner (Brilliance iCT 256, Philips Healthcare), cerebral and cervical CTA examinations were performed from the aortic arch, and the parameters were the field of view = 220 mm, tube voltage = 120 kVp, tube current = 300 mAs, and the slice thickness = 1 mm. Bolus tracking technique was used with a 20 ml saline bolus followed by 50 ml Iohexol (Omnipaque 350, GE Healthcare) and a 20 ml saline bolus with a 5 ml/s injection rate. With the help of the postprocession workstation (IntelliSpace Portal), these arteries were reconstructed and evaluated. Final decisions were made on the thin section images.

The article "Relationship between Circle of Willis Variations and Cerebral or Cervical Arteries Stenosis Investigated by Computer Tomography Angiography and Multitask Convolutional Neural Network" was published in 2021. Journal: J Healthc Eng.

### 2.3. Assessment of the CoW and Arteries Stenosis

Each segment of the CoW was classified as “normal” or “variation.” The segment that could not be visualized in CTA images was defined as a variation. It should be noted that due to a lack of consensus for the definition of hypoplasia, the precommunicating part of the anterior cerebral artery (A1), precommunicating part of the posterior cerebral artery (P1), or posterior communicating arteries (Pco) with diameters over 70% thinner than contralateral segments were also classified as “variation.” Even though it was not shown clearly, the anterior communicating artery (Aco) should be classified as “normal” in case of the bilateral ACAs being fused. Then, the entire CoWs, both anterior and posterior parts, were considered separately and classified as complete (all segments normal) and incomplete (any of the segments exhibiting a variation).

The degree of arterial stenosis, including CCA, ICA, BA, VA, and major branches of cerebral arteries, was determined according to the criteria established by the North American Symptomatic Carotid Endarterectomy Trial (NASCET) and categorized into “normal,” “mild stenosis” (≤29%), “moderate stenosis” (≥30% and ˂70%), and “severe stenosis” (≥70%).

### 2.4. Statistical Methods

Each subject was assessed by two independent radiologists (R1 with 17 years of experience in vascular imaging; R2 with 5 years of experience). In case of discrepancy, an agreement was reached by consensus. GraphPad Prism version 5.1 and SPSS 20.0 were used for statistical analysis. Comparisons between groups were conducted using the *t*-test or chi-square test where appropriate, with *P* < 0.05 considered statistically significant. All the tests were not corrected for multiple comparisons.

### 2.5. Datasets and Preprocessing

30 CTA datasets were selected and manually delineated as ground truth using the Mimics V17. We divided them into a training group (24 cases) and a validation group (6 cases). Furthermore, we collected another 61 datasets as a testing group. Isotropic resampling was firstly adopted to generate datasets with the same spacing of 0.5 mm in the *x*-*y*-*z* directions. Then, thresholding was used to exclude the interference of background voxels with an intensity lower than 0 or higher than 2000.

### 2.6. The Proposed Model

A multitask CNN model was proposed, and its architecture is shown in Figure 1.

Multitask models have been proven their effects in different deep learning tasks [17]. We adopted the multitask idea to propose a multitask CNN for cerebral vessel segmentation. We formatted the CTA image as a weighted summation of the background and foreground (vessels). The weight map could be considered as the segmentation probability. The proposed model has one input and three output heads to simultaneously reconstruct the background, foreground, and weight map. We constructed a reconstruction loss to evaluate the dissimilarity between the input image and output reconstruction image, which is the weighted summation of background and foreground image. We also added a segmentation loss to evaluate the difference between the weight map and vessel ground truth segmentation. The summation of reconstruction loss and segmentation loss is used as the multitask loss function to optimize the proposed model.

The article "Relationship between Circle of Willis Variations and Cerebral or Cervical Arteries Stenosis Investigated by Computer Tomography Angiography and Multitask Convolutional Neural Network" was published in 2021. Journal: J Healthc Eng.

The proposed network adopted an encoder-decoder structure with multihead output. An atrous spatial pyramid pooling (ASPP) module was used to merge multiscale high-level features to enhance the recognition power of small-sized objects. The multihead output consisted of two reconstruction outputs and a segmentation output, which were used to compute the multitask loss function. The multitask loss function was helpful to produce a model with higher generalization ability.

The model adopted an encoder-decoder structure. The encoder network employed 4-level convolutions with a kernel size of 3 and max-pooling to extract high-level features. The extracted high-level features were sent to an atrous spatial pyramid pooling to concatenate multiscale features generated by global average pooling and parallel convolution with dilation rates of 1, 2, 4, and 8. Then, a decoder network was used to recover spatial information by upsampling operations and skipping connections, which concatenate low-level features and high-level features together. Finally, three branches were connected to generate 3 different outputs, including the segmentation probability map *O*, the reconstructed foreground *F*, and the background *B*. Two tasks were involved in the model: the reconstruction task and the segmentation task. We then built a multitask loss function for model optimization as follows:

(1) $$\begin{array}{c} J\left(\theta |I,S\right)=\frac{1}{N}\sum_{i=1}^{N}{\left(I_{i}-\left(F_{i}*O_{i}+B_{i}*\left(1-O_{i}\right)\right)\right)}^{2}+\frac{1}{N}\sum_{i=1}^{N}\left(1-2*\frac{O_{i}*S_{i}}{O_{i}^{2}+S_{i}^{2}}\right), \end{array}$$

where *I* and *S* are training image and respecting ground truth, *N* is the number of training images, and *θ* represents the model parameters. The first term is the reconstruction loss, which computes the mean squared error between the input and the reconstructed images. The reconstructed image is a weighted summation of the foreground *F* and the background *B* with probability *O* as weights. The second term computes the Dice loss between ground truth *S* and probability map *O* to evaluate the loss of segmentation.

The article "Relationship between Circle of Willis Variations and Cerebral or Cervical Arteries Stenosis Investigated by Computer Tomography Angiography and Multitask Convolutional Neural Network" was published in 2021. Journal: J Healthc Eng.

During training, axial slices of 288 × 288 were extracted from CTA training images and augmented by rotation and flipping. We used Adam optimizer with an initial learning rate of 0.0001. The model is trained by 50 epochs with a batch size of 32.

### 2.7. Model Evaluation

The Dice coefficient (DC) was employed as the metric to evaluate the segmentation accuracy of the model on the validation group. The 61 datasets of the testing group were segmented by the model, and the segmentation accuracy was evaluated in the labelled images.

## 3. Results and Discussion

### 3.1. General Characteristics and the Prevalence of Variations of CoW

255 cases were included (160 males, mean age 57 ± 17 years, range 21–84 years). The characteristics are shown in Table 1, classified by age and degree of stenosis. Of these, some cases from “afferent + mild stenosis” and “afferent + moderate stenosis” were categorized into an “AMs” group, and some cases from “young + normal,” “senior + normal,” and “afferent + mild stenosis” were categorized into an “Ec” group.

Figure 2 demonstrates the prevalence of variations of CoW reported by the previous and present imaging-modality studies [18].

### 3.2. Variations of Individual Segments and the Completeness of the CoW in Different Populations

The prevalence of the variations of the individual segments and the completeness of CoW is demonstrated in Table 2. Sex has been matched between Yn and Sn. The prevalence of variation of Aco and incompleteness of the anterior part of the CoW was significantly higher in Sn than in Yn (*P*=0.046 and 0.009, respectively). Age has been matched between males and females, and the prevalence of the variation of Aco and incompleteness of the anterior part of the CoW was higher in females than in males (*P*=0.024 and 0.044, respectively). Both sex and age had been matched among Sn, AMs, and Ass, and between ESs and Ec. Patients with stenosis of the afferent and efferent arteries did not exhibit a significant change in the prevalence of variation of individual segments and the incompleteness of the CoW.

### 3.3. Results from the Proposed Deep Learning Model

#### 3.3.1. DC Evaluates the Overlap between the Prediction *O* and Ground Truth *F*

(2) $$\begin{array}{c} \text{DC}=\frac{2*\left|O*F\right|}{\left|O\right|+\left|F\right|}. \end{array}$$

A greater DC value (close to 1) means better segmentation. DC will be 0 if the prediction and ground truth have no overlap. The complete cerebral and cervical arteries could be segmented and reconstructed in 120 s, and an average DC of 78.2% was achieved by the proposed multitask model. We also trained a single-task U-Net model for comparison, which only involved the segmentation task without reconstruction. The average DC of the single-task model was 74.3%, nearly 4% lower than the proposed model. The results indicate that multitask learning can help enhance feature discrimination and improve generalization ability.  Figure 3 shows the segmentation results of the proposed multitask model and single-task model. The results suggest that the proposed model can generate better segmentation in thinner vessel areas with less noise than a single-task model.

The article "Relationship between Circle of Willis Variations and Cerebral or Cervical Arteries Stenosis Investigated by Computer Tomography Angiography and Multitask Convolutional Neural Network" was published in 2021. Journal: J Healthc Eng.

#### 3.3.2. The Accuracy of the Model Visually Evaluated by Experts

Using the proposed model and head-neck CTA data, the segmentation accuracy for P1 was determined to be perfect at 100%, and A1 and Pco were 99.2% and 94%, respectively, while for Aco, the accuracy significantly decreased to 69% (Figure 4).

### 3.4. Discussion

Compared with the Aco and anterior part of the CoW, the higher prevalence of Pco variation and incompleteness of posterior circle were demonstrated in both young and senior normal populations. It may be correlated with their functional significance. Aco is considered the most important collateral pathway and helps retain blood flow in the cerebral hemispheres [19]. Thus, its absence or hypoplasia will be more costly in cerebrovascular events Pco. However, the prevalence of Pco variation reported from the imaging study was different from the dissection study. Using imaging methods, the prevalence of hypoplasia of the Pco ranges from 23% to 41%, and the prevalence of absence of the Pco ranges from 22% to 48% while in dissection, the hypoplasia of the Pco has a prevalence of 23–70% and is absent 0%–14% of the time. A higher prevalence of absence in imaging studies may be related to a lower spatial resolution of this technique. The maximum spatial resolution of CTA is 0.14 mm, while in dissection, the arteries with diameters less than 0.1 mm can be observed [20, 21].

We also demonstrated that the values of the prevalence of variation and incompleteness were generally more prominent than those reported in the literature. This could be attributed to several factors. The definition of “variation” was different between studies. In our study, the variation was defined as nonvisualization in CTA images or diameters over 70% thinner than contralateral segments, which might include both absence and hypoplasia observed in previous studies. Moreover, racial differences could partly contribute to the high prevalence [22]. Compared to Westerners and Japanese populations, a higher prevalence of an incomplete posterior portion of the CoW has been reported in the Chinese populations [23].

The article "Relationship between Circle of Willis Variations and Cerebral or Cervical Arteries Stenosis Investigated by Computer Tomography Angiography and Multitask Convolutional Neural Network" was published in 2021. Journal: J Healthc Eng.

A major finding is that neither the stenosis of afferent arteries nor the stenosis of efferent arteries affects the configuration of the CoW. Dissection is not suitable for such research directed at the association of the CoW with diseases because it is hard to differentiate healthy individuals from patients, so *in vivo* imaging techniques have been employed to facilitate such studies. Waaijer et al. found that a compromised anterior circle segment was detected more frequently in patients with symptomatic carotid artery stenosis than in controls [24]. Hartkamp found a higher percentage of complete CoW in patients (55%) with ICA stenosis than in normal (36%) [25]. Varga assessed the CoW of 544 patients with severe stenosis of the ICA and suggested that ICA stenosis was the only independent predictor of CoW configuration [3]. The differences between our results and previous reports may be due to the age and sex of the subjects. To date, most studies suggest that the variations or anomalies demonstrated in the fetal period continue into postnatal life and age-related segment changes only arise if lesions occur.

Moreover, no significant gender differences in the prevalence of variations have been observed in almost all studies [5, 23, 26, 27]. The matching of age or sex was seldom performed in previous studies that investigated the influence of stenosis on CoW variation. Our results demonstrate a significant association between CoW variation and age or gender and suggest that possible biases arise unless the age and gender are matched among groups. Moreover, the possible reasons for these variations are suggested. Two factors are thought to play important roles: gene and hemodynamics. The latter is related to the degeneration of embryo arteries, the functional significance of vascular segments, neck movement, and the presence of pathological lesions [19, 26, 28]. In Vasovic's words, it is “a theoretical model in prenatal and postnatal developmental phases” [29]. Our result suggests that crucial factors for variation favor genetic and physiological factors over hemodynamics changes resulting from pathological lesions. However, although differences were not statistically significant, there was a noted tendency toward a lower prevalence of variation of the P1 in patients with severe stenosis of efferent arteries, so a larger sample size is necessary to verify the opinion. Another limitation is that the data of this study were collected from only one institution, and the results need more verification in other institutions.

It was exciting that, with the help of a deep learning model, CoW could be quickly segmented and reconstructed with high DC. In contrast, it would take an experienced radiologist more than 1 hour to manually delineate complete cerebral and cervical arteries. The performance of the model was perfect for segmenting P1, A1, and Pco, but it should be improved in Aco. The vessel would not be accurately discriminated and segmented if its diameter was less than 3 mm, and the absence of Aco would not be recognized if bilateral ACA were too close. Even more noteworthy was that the visual-evaluation results from 7 cases were revised and improved with the aid of AI. So, the deep learning-based method can increase the efficiency of brain vessel segmentation and improve the accuracy of visual evaluation by a radiologist.

The article "Relationship between Circle of Willis Variations and Cerebral or Cervical Arteries Stenosis Investigated by Computer Tomography Angiography and Multitask Convolutional Neural Network" was published in 2021. Journal: J Healthc Eng.

However, the segmentation performance is still suffering from the following limitations. (1) Only limited labelled datasets are used for model optimization, leading to low generalization ability. Future work would include semisupervised segmentation models that employ limited labelled datasets and more unlabelled datasets for training [30, 31]. (2) The proposed model performs worse in detail, particularly discriminating between closely associated vessels and small-sized vessels, which is a typical problem in other medical image analysis tasks [32].

## 4. Conclusions

The study suggests that key factors for variation of CoW favor genetic and physiological factors over hemodynamics changes resulting from pathological lesions. A multitask CNN model is developed to segment CoW automatically, and its performance is validated in the diagnosis of the variation. It can be considered an adjunct tool for investigating the variation, particularly related to reducing workload and improving the accuracy of the visual evaluation.

## Figures and Tables

**Figure 1:** The architecture of the proposed multitask segmentation method.

**Figure 2:** Schematic drawing labelled with the prevalence of absence of each segment of the Cow and incompleteness of the anterior and posterior circle from the present and previous imaging-modality studies. pACA: postcommunicating part of an anterior cerebral artery; A1: precommunicating part of an anterior cerebral artery; Aco: anterior communicating artery; pMCA: postcommunicating part of a middle cerebral artery; ICA: internal carotid artery; Pco: posterior communicating arteries; P1: precommunicating part of a posterior cerebral artery; pPCA: postcommunicating part of a posterior cerebral artery; BA: basilar artery.

**Figure 3:** Results of segmentation and reconstruction. (a) One axial CTA slice labelled manually by an experienced radiologist and 3D meshes of ground truth. (b) One axial CTA slice segmented by the proposed model and the 3D meshes. (c) One axial CTA slice segmented by the single-task model and the 3D meshes. Comparison with a single-task model (c); more details, which were highlighted in an oval in (b), can be shown using the proposed multitask model.

The article "Relationship between Circle of Willis Variations and Cerebral or Cervical Arteries Stenosis Investigated by Computer Tomography Angiography and Multitask Convolutional Neural Network" was published in 2021. Journal: J Healthc Eng.

**Figure 4:** Wrong segmentation based on the proposed model for CoW. (a) Close bilateral ACA was wrongly delineated together and considered as Aco, which is a most common error. (b) Right A1 was not completely delineated. (c) Right Pco was not delineated. (d) Another vessel was wrongly delineated as Pco.

**Table 1:** Characteristics of patients.

Group	Cases	Age (y) (mean ± SD)	Male (%)
Young + normal	53	30 ± 4	68
Senior + normal	41	61 ± 5	34
Afferent + mild stenosis	55	71 ± 6	56
Afferent + moderate stenosis	24	67 ± 6	67
Afferent + severe stenosis	34	68 ± 9	76
Efferent + severe stenosis	48	51 ± 13	77

Patients were categorized according to age and the severity of cerebral carotid artery stenosis. “Young + normal” refers to patients aged 21–35 years without stenosis of an artery; “senior + normal” refers to patients aged 55–76 years without stenosis of an artery; “afferent” refers to the arteries including CCA, ICA, BA, and VA. “Efferent” refers to the arteries, including the postcommunicating parts of ACA, MCA, and PCA. The degree of stenosis of arteries was determined according to the criteria of NASCET and categorized into “normal,” “mild” (≤29%), “moderate” (≥30% and ˂70%), and “severe” (≥70%).

**Table 2:** Prevalence of variation in individual segments and incompleteness in the CoW.

Group	Cases	Ages (y)	Male (%)	Variation (%)				Incompleteness of CoW (%)		
				Aco	A1	Pco	P1	Entirety	Anterior part	Posterior part
*Group 1 divided according to age*										
Yn	53	30 ± 4	68	36^*∗*^	11	85	25	98	47^*∗*^	96
Sn	27	63 ± 5	48	59^*∗*^	22	96	15	100	78^*∗*^	96

*Group 2 divided according to sex*										
Male	40	42 ± 15	100	30^*∗*^	10	93	18	100	40^*∗*^	98
Female	40	48 ± 15	0	55^*∗*^	18	90	23	95	63^*∗*^	93

*Group 3 divided according to afferent arteries stenosis*										
AMs	41	66 ± 6	61	49	12	95	10	98	61	98
ASs	27	67 ± 9	74	48	22	93	19	100	67	96

*Group 4 divided according to efferent arteries stenosis*										
ESs	50	51 ± 13	78	32	24	88	8	94	52	84
Ec	65	53 ± 16	68	40	17	86	20	97	56	94

Group 1: sex has been matched between Yn and Sn. ^*∗*^The prevalence of variation of Aco and incompleteness of the anterior part of the CoW was significantly higher in Sn than in Yn (*P*=0.046 and 0.009, respectively). Yn: young normal group (Yn), those aged 21–35 years without stenosis of an artery. Sn: senior normal group (Sn), those aged 55–76 years without stenosis of an artery. Group 2: age has been matched between males and females. ^*∗*^The prevalence of the variation of Aco and the incompleteness of the anterior part of the CoW was higher in females than in males (*P*=0.024 and 0.044, respectively). Group 3: both the age and sex had been matched among Sn, AMs, and ASs. Patients with stenosis of the afferent arteries did not exhibit a significant change in the prevalence of variation of individual segments and the incompleteness of the CoW. AMs: mild-moderate stenosis group in afferent arteries group with mild-moderate stenosis of CCA, ICA, or BA but without simultaneous severe stenosis of VA. ASs: severe stenosis in afferent arteries group, those with severe stenosis of CAA, ICA, BA, or bilateral VA. Group 4: both the age and sex had been matched. There was a lower prevalence of variation of P1 segment and incompleteness of the posterior part in ESs than in Ec with no significant difference (*P*=0.072 and 0.087, respectively). ESs: severe stenosis of efferent arteries group with severe stenosis of postcommunicating parts of ACA, MCA, or PCA, and normal or middle stenosis of afferent arteries. Ec: control group of ESs, those with normal postcommunicating parts and normal or middle stenosis of afferent arteries.

The article "Relationship between Circle of Willis Variations and Cerebral or Cervical Arteries Stenosis Investigated by Computer Tomography Angiography and Multitask Convolutional Neural Network" was published in 2021. Journal: J Healthc Eng.

## Data Availability

The data used to support the findings of this study are available from the corresponding author upon request.
